This article has been retracted.

# The Application Value and Influence of Integrated Nursing of Operating Room and Disinfection Supply Center Combined with 6Sigma Management in Operating Room Instruments

**DOI:** 10.1155/2022/8490473

**Published:** 2022-08-16

**Authors:** Xiaomin Zhu, Ying Xu, Xuefei Hu, Hong Ye, Jun Xiao

**Affiliations:** ^1^Wuhan First Hospital Operating Room, 430022, China; ^2^Orthopedic Trauma Department, Wuhan Fourth Hospital, 430033, China

## Abstract

In this study, 897 surgical instruments used for comprehensive management of hand supply from January to December 2019 were selected as the control group. Similarly, 1086 surgical instruments administered with 6Sigma from January to December 2020 were selected as the observation group. By observing and comparing the differences between the two groups of patients in the operating room equipment cleaning pass rate and general indicators, other related pass rate, operating room equipment defects, and doctors' satisfaction with equipment, to explore the application value and influence of comprehensive nursing in operating room and disinfection supply center combined with 6Sigma management in operating room equipment management. The results show that the application of hand-supply integration combined with 6Sigma management has a good effect on operating room equipment management, which significantly improves the qualified rate of operating room equipment cleaning and the satisfaction of doctors to the equipment, and reduces the defects of operating room equipment, which has a certain reference value for operating room equipment management.

## 1. Introduction

As one of the core departments of a hospital, the operating room undertakes surgical treatment tasks in all departments of the hospital and is closely related to patients' lives [1]. With advances in medical science and technology, the development of surgical techniques quickly, intensity of the use of operating frequency, the type of surgery, surgery, and surgical instrument classification also will increase, followed by surgery work involved in a wider range and surgical instruments; the management difficulty increases; thus, operating room rate of adverse events due to equipment management was increased; the protection of the operating room and the refinement and specialization of the division of labor put forward higher requirements, requiring medical staff to strengthen the integrated device management of surgical instruments and disinfection supply center [2, 3].

The 6Sigma model [4] was first put forward by Motorola engineers, dedicated to the pursuit of work quality and efficiency and is a kind of including the definition, measurement, analysis, improvement, and process control; through the set goals, collect the data; the results of the analysis, in order to reduce the defects of products and services, establish a high-quality and efficient management system. This management system strictly controls the device preparation process to ensure patient safety and comfort during surgery [5]. Operating room instrument management refers to centralizing the used instruments in the supply room for inventory, inspection, cleaning, maintenance, disinfection, and sterilization, returning the instruments to the operating room for use, ensuring the normal supply of daily operations, and effectively integrating with the 6Sigma model, a set of practical workflow and management mode [4]. Based on this, our hospital has conducted a certain exploration to explore the application value and impact of the integration of operating room and disinfection supply center combined with 6Sigma management in operating room equipment management. The current research results are reported as follows.

## 2. Materials and Methods

### 2.1. General Information

Selected from January to December 2019, 897 surgical instruments were used for integrated management of hand supply as the control group, including 165 skin hooks, 216 tissue forceps, 196 hemostatic forceps, 145 S hooks, and 126 needle holders. Pieces: there are 49 pieces of cavity mirrors. In the same way, 1086 surgical instruments used for the implementation of 6Sigma management from January to December 2020 were selected as the observation group, including 330 tissue forceps, 230 hemostatic forceps, 142 S-shaped hooks, 147 needle holders, and 137 cavities mirror. The operating room and the disinfection supply room have little change in personnel and are comparable (Figure 1).

### 2.2. Method

The control group adopted integrated management of hand-supply equipment in the operating room, that is, the operating room was specially equipped with 2 nurses to inspect and pack the equipment in the supply room, and the supply room was equipped with 2 nurses to inspect and pack the equipment in the operating room. After each operation, the instrument nurse sends the instruments after the operation to the washing room and rinses the stains and blood on the surface of the instruments with tap water. The processed instruments are arranged before packaging, and all instruments with shaft joints are opened. After two people check the base number and sign, they are put into a special instrument basket. The assembled instrument basket is placed in a plastic storage box for storage. If it is a surgical instrument with a special infection, the instrument nurse should soak the surgical instrument in 500 mg/L chlorine-containing disinfectant for 30 minutes, then treat it according to the above requirements, and use a red prescription to indicate the type of infection. 34 times a day, the staff in the supply room must collect surgical instruments in the operating room at a fixed time to complete the receipt and delivery of the instruments. The staff in the blood supply room perform a series of standardized processes such as cleaning, enzymatic washing, ultrasonic oiling, drying, inspection, packaging, and disinfection of the surgical instruments and then send the sterilized surgical instrument packs to the operating room and the equipment team in the operating room. The nurse handed over and signed for. If the equipment has quality problems, the general equipment will be replaced by the supply room, and the special equipment will be replaced by the operating room.

The observation group implemented 6Sigma management on the basis of the control group, that is, (1) definition: set up 6Sigma intervention group, which is composed of the nursing director, the head nurse of the big department, the head nurse of the disinfection supply center, the head nurse of the operating room, the disinfection supply center, and the group leader of the operating room subspecialty. All of them have gone through systematic 6Sigma lean training, and the director of the nursing department is responsible for the management and work arrangement of the group; this stage is mainly to clarify the problems existing in modular classification management, how to improve the restriction steps of modular classification management, and how to implement the modular management to speed up the handover of operating room and instrument room, aiming at the above problems to develop goals to be achieved, through 6Sigma management to strengthen the quality control of the management process. (2) Evaluation: this stage is mainly to analyze the problem, with the help of the present stage department narrow the scope of the problem of critical data, clear the key problems in the process of equipment management, analyze the core of the problem, record the amount of surgical instruments, current equipment cleaning and disinfection qualified rate, equipment fault rate, and other data, and determine the problems be solved in the course of equipment management and instruments such as speeding up the operating room. The factors affecting the handover between rooms can be evaluated according to the sequence of processes. (3) Analysis: the methods of observation method, interview method, and logic method, an analysis of the causes of the problems caused by using fishbone diagram to confirm causal relationship, in the form of list's current operation process, and according to the people (staff), machine (machine), materials (material), law (law), ring (environment), and so on, factors affecting the selection of surgical instrument management in each step one by one, all that affect the phase. For example, it is easy to be damaged or lost in the transfer process due to improper operation of personnel, insensitive electronic entry system, different shapes and sizes of instruments, etc., whether the rules and regulations of the department for noninstrument handover are scientific, reasonable, and comprehensive, and the distance between the operating room and the instrument supply room is too far for handover, etc. (4) Improvement: to summarize all the influencing factors and targeted development of improvement plan. For example, in the case of nonstandard operation and easy omission, personnel training should be strengthened, and the use table of devices should be made to track and record the use department, personnel, time, number of pieces, and return of each device. In order to improve the equipment cleaning process, personnel in the disinfection supply center can be reassigned, and the amount of surgical instruments used during peak hours can be reasonably arranged and decomposed, and humanized shift system can also be adopted. Strengthen the use of information center management system and seamless connection of the disinfection supply center; all equipment storage, use, docking, cleaning, disinfection, sterilization, and other processes should be recorded into the system, in order to trace and track the quality and expiration date of disinfection items and personnel situation. (5) Control: according to the specific method in the improvement system, determine the control standard, for the problems in the improvement, which should be timely reported to the management responsible person; discuss solutions, to avoid the occurrence of big mistakes. In order to standardize the rules and regulations, the responsibilities of all nursing personnel should be clearly defined in the operation process, and the quality control of each link should be strengthened to ensure that the quality of equipment reaches the standard. The management personnel shall also complete the quality assessment of the responsible nurses every month and monitor and evaluate the preoperative preparation, intraoperative use, postoperative treatment, and storage of surgical instruments of the nurses during perioperative period.

### 2.3. Statistical Methods

The data in this study was calculated using Excel and reviewed by two physicians. The selected data are in accordance with the normal distribution. After the first author and corresponding author have entered the data into the computer system and proofread, the statistical software is used for SPSS25.0 to perform related calculations. The count data expressed in percentage (%) or integer were tested by *χ*^2^, and statistical *P* < 0.05 indicated that the difference was statistically significant.

## 3. Result

### 3.1. Comparison of Qualification Rate of Equipment Cleaning in Operating Room

The qualified rate of tissue forceps, hemostatic forceps, S hook, needle holder, and endoscope in the observation group was higher than that in the control group, and the difference was significant (*P* < 0.05) (see Table 1).

### 3.2. Comparison of Other Relevant Qualification Rates

Observation group's operating room equipment had a higher level of qualified sterilization, loss and wastage, qualified item packaging, equipment damage, and late delivery of equipment than those of the control group, which was statistically significant (*P* < 0.05) (see Table 2).

### 3.3. Comparison of Equipment Defects in Operating Room

Observation group's improper placement, unregistered after use, not repaired in time, unmatched parts, incomplete preparation, and poor function were significantly lower than those of the control group. The difference was statistically significant after testing (*P* < 0.05) (see Table 3).

### 3.4. Physician's Satisfaction with the Device

The 99.63% of physicians' satisfaction with observation group's devices was significantly higher than that of control group's 96.10%. There was no significant difference in the chi-square test (*P* > 0.05) (see Table 4).

## 4. Discussion

Operating room is an important link in the hospital; each department maintains normal operation; disinfection supply center is the key to the auxiliary operating room efficient operation departments, to realize the integration of the operating room—disinfection supply center system, surgical instruments equipped with scientific and standardized management system is a modern operating room—and disinfection supply center runs irreversible trend [6]. The application of appropriate management methods in the operating room-disinfection supply center integration system is an effective guarantee for improving the quality of treatment and nursing, optimizing personnel allocation, reducing the incidence of adverse events, and improving the comprehensive strength of the hospital [7]. 6Sigma intervention was first proposed by Motorola engineers. It is a management strategy used to improve enterprise quality and optimize process management. It takes setting objectives, receipt data, and analysis results as the means to achieve “zero defect” and aims to improve quality and reduce cost [8]. At present, lean 6Sigma technology has been applied in various fields and enterprises and achieved excellent results. Some scholars [9] applied the 6Sigma management method to the management of operating room instruments and equipment, which had significant effects on improving the completeness rate of operating room instruments and equipment, shortening the preparation time before the use of instruments and equipment, and improving the satisfaction of surgeons. Modular classification is a specific embodiment of the integrated management system of operating room and disinfection supply center, which classifies surgical medical instruments according to their needs, facilitating tracking, use, and sorting, realizing reasonable allocation of resources, and improving the work efficiency of nursing staff in disinfection supply center [10]. The combination of 6Sigma and modular classification can make the operation room and disinfection supply center more efficient and high quality, and its clinical application value can be seen.

Hand-supply integration can effectively avoid problems such as improper maintenance of surgical instruments and poor disinfection quality due to insufficient professional training in surgery and inadequate technical updates and effectively improve the management level of surgical instruments [6]. However, in the specific implementation process, it was found that there are still some shortcomings in the integrated management of hand-supply [11]. Therefore, in the implementation of hand-supply integration, certain interventions are needed to reduce and eliminate various drawbacks [7]. Thereby, improving the use effect of surgical instruments is also an important basis for improving the cleaning quality and disinfection effect of surgical instruments [8]. The use of 6Sigma management mode realizes the continuity of surgical instruments from the recovery and supply to clinical application, makes the management process of surgical instruments more scientific and reasonable, and improves the cleaning and disinfection quality of surgical instruments [9, 10, 12, 13]. Professional cleaning is conducive to the professional protection of full-time personnel in the disinfection supply center and is compatible with the degree of specialization, specialization, and mechanization of the full-time personnel in the disinfection supply center [10, 12]. The 6Sigma management model effectively regulates the use, classification, and operating standards of nurses in the nursing operating room and disinfection supply room through stage training and improves the organization and project management techniques of nurses in the nursing operating room and disinfection supply room [13–15].

This study explored the application of hand-supply integration and 6Sigma management in operating room equipment management. The results showed that the observation group's operating room equipment's qualified sterilization, loss, and wastage and qualified item packaging, equipment damage, and late delivery of equipment were significantly higher than that in the control group; the observation group's improper placement, unregistered after use, failure to repair in time, unmatched parts, incomplete preparation, and poor function were significantly lower than those in the control group. The doctor's satisfaction with the observation group's equipment was significantly higher than 99.63% and 96.10% of the control group. It shows that the application of hand-supply integration combined with 6Sigma management in operating room equipment management has a better effect, significantly improving the qualification rate of operating room equipment cleaning and physicians' satisfaction with equipment and reducing operating room equipment defects. Strictly standardize equipment recycling, cleaning, sterilization, maintenance, and supply, ensure equipment quality and equipment management practices, evaluate problems in the management process, analyze the factors affecting the problem, determine the core and goal of solving the problem, optimize the nursing process, and improve nursing quality [16–20]. The management of surgical instruments in the disinfection supply center can avoid the purchase of duplicate equipment in the operating room and can also reduce the nonnursing work time of the nurses in the operating room, which is conducive to reducing pollution and rational use of resources, reducing the number of times the operating room staff come into contact with contaminated instruments, and reducing operation chances of contaminated employees [21–24].

The 6Sigma management model is a new quality control model, which can realize continuous quality control of surgical instruments from recovery and supply to clinical application [25–29], to ensure that the surgical instrument management process is more scientific and to further ensure the quality of instrument disinfection, reduce the work pressure of nurses, improve work efficiency, and increase physician satisfaction [30, 31]. In the process of hand-held integrated surgical instrument management, the 6Sigma management mode uses phase control such as clarification, evaluation, analysis, improvement, and control to discover problems in instrument management in a timely manner [32]. Formulating reasonable improvement measures, perfecting the management system, rationally deploying personnel and equipment, effectively reducing the labor intensity of nursing staff in the operating room, and ensuring the quality of equipment cleaning are of great significance for improving the quality of care [33–35]. The application of the 6Sigma management model can help reduce the loss and loss of equipment, improve the qualification rate of packaging and sterilization, and significantly improve the satisfaction of doctors with nursing work, which is worthy of clinical promotion.

In summary, the application of hand-supply integration combined with 6Sigma management in operating room equipment management has a better effect, significantly improving the qualification rate of operating room equipment cleaning and physicians' satisfaction with equipment, reducing operating room equipment defects, and having a certain effect on operating room equipment management reference value.

## Figures and Tables

**Figure 1:** The research procedure.

**Table 1:** Comparison of the qualification rate of equipment cleaning in the operating room between the two groups [*n* (%)].

Group	Tissue forceps qualification rate	Qualified rate of hemostatic forceps	S hook qualification rate	Qualified rate of needle holder	Qualification rate of cavity mirror
Control group (897)	206 (95.37)	162 (82.65)	126 (86.90)	113 (89.68)	37 (75.51)
Observation group (1086)	319 (96.67)	211 (91.74)	139 (97.89)	141 (95.92)	132 (96.35)
*χ* ^2^	4.417	4.235	4.079	32.810	139.501
*P*	0.031	0.032	0.039	0.000	0.000

**Table 2:** Comparison of other relevant qualification rates [*n* (%)].

Group	Sterilization qualification rate	Loss attrition rate	Goods packaging qualification rate	Equipment damage rate	Late delivery rate of equipment
Control group (897)	886 (98.77)	862 (96.10)	126 (14.10)	793 (88.41)	787 (87.74)
Observation group (1086)	1082 (99.63)	1061 (97.70)	119 (10.96)	1071 (98.61)	1079 (99.36)
*χ* ^2^	4.817	4.285	4.329	87.462	117.693
*P*	0.028	0.031	0.037	0.000	0.000

**Table 3:** Comparison of equipment defects in the operating room between the two groups [*n* (%)].

Group	Inappropriate placement	Not registered after use	Not repaired in time	Parts are not matched	Not ready	Poor function
Control group (897)	22 (24.53)	49 (54.63)	32 (35.67)	27 (30.10)	25 (27.87)	19 (21.18)
Observation group (1086)	13 (11.97)	12 (11.05)	16 (14.73)	18 (16.57)	14 (12.89)	8 (7.37)
*χ* ^2^	4.467	29.899	9.121	4.052	5.717	6.981
*P*	0.035	0.000	0.003	0.044	0.017	0.008

**Table 4:** Two groups of physicians' satisfaction with devices [*n* (%)].

Group	Very satisfied	Satisfy	Generally	Dissatisfied	Satisfaction
Control group (897)	640	122	100	35	862 (96.10)
Observation group (1086)	582	230	270	4	1082 (99.63)
*χ* ^2^	/	/	/	/	31.814
*P*	/	/	/	/	0.000

## Data Availability

No data were used to support this study.

## References

[1] Bruner E., Fedato A., Silva-Gago M. (2019). Visuospatial integration and hand-tool interaction in cognitive archaeology. *Current Topics in Behavioral Neurosciences*.

[2] Yalachkov Y., Kaiser J., Doehrmann O., Naumer M. J. (2015). Enhanced visuo-haptic integration for the non-dominant hand. *Brain Research*.

[3] Prsic A., Boyajian M. K., Snapp W. K., Crozier J., Woo A. S. (2020). A 3-dimensional-printed hand model for home-based acquisition of fracture fixation skills without fluoroscopy. *Journal of Surgical Education*.

[4] Pang C., Li H., Luo L., Wang X. (2020). Application of 6Sigma management method to improve the effect of hospital scientific research management. *Chinese Journal of Medical Science Research Management*.

[5] Wenxia L., Yuhong L., Weili Z. (2020). Application of six sigma management model in orthopedic robotic surgery training for new nurses. *Chinese Journal of Modern Nursing*.

[6] Qu H., Xu Y. (2020). Development and application of surgical implant traceability system based on hand-supply integration. *Chinese Journal of Modern Nursing*.

[7] Wang J. (2017). The impact of PDCA quality control circle on the integrated management of operating room and supply room. *Medical and Health Equipment*.

[8] Yan L. (2017). The application value of quality control circle in the integrated management model of operating room and supply room. *Chinese Journal of Woman and Child Health Research*.

[9] Liu H., Zhang X., Li J. (2019). Band and phonon engineering for thermoelectric enhancements of rhombohedral GeTe. *ACS Applied Materials & Interfaces*.

[10] Hickey E. J., Halvorsen F., Laussen P. C., Hirst G., Schwartz S., van Arsdell G. S. (2018). Chasing the 6-sigma: drawing lessons from the cockpit culture. *The Journal of Thoracic and Cardiovascular Surgery*.

[11] Caixia S., Guo Y., Zheng H. (2020). The influence of "integration of hand-supply" on equipment management in operating room. *Chinese Medicines and Clinics*.

[12] Lee K. L. K., McCarthy M. (2019). Study of benzene fragmentation, isomerization, and growth using microwave spectroscopy. *Journal of Physical Chemistry Letters*.

[13] Zhang X. Y., Guo J. C. (2020). Dynamic fluxionality of ternary Mg2BeB8 cluster: a nanocompass. *Journal of Molecular Modeling*.

[14] Krajewski L. C., Rodgers R. P., Marshall A. G. (2017). 126 264 assigned chemical formulas from an atmospheric pressure photoionization 9.4 T Fourier transform positive ion cyclotron resonance mass spectrum. *Analytical Chemistry*.

[15] Wang Y. J., Feng L. Y., Xu L. (2020). Boron-based ternary Rb6Be2B6 cluster featuring unique sandwich geometry and a naked hexagonal boron ring. *Physical Chemistry Chemical Physics*.

[16] Formaggio J. A., Kaiser D. I., Murskyj M. M., Weiss T. E. (2016). Violation of the Leggett-Garg inequality in neutrino oscillations. *Physical Review Letters*.

[17] Wang Y. J., Guo M. M., Wang G. L., Miao C. Q., Zhang N., Xue T. D. (2020). The structure and chemical bonding in inverse sandwich B6Ca2 and B8Ca2 clusters: conflicting aromaticity vs. double aromaticity. *Physical Chemistry Chemical Physics*.

[18] Feng L. Y., Wang K., Zhai H. J. (2020). Anchoring a bow-shaped boron single chain in binary Be6B7- cluster: hybrid octagonal ring, multifold *π*/*σ* aromaticity, and dual electronic transmutation. *Physical Chemistry Chemical Physics*.

[19] Chen H., Guo Y., Wei H. (2020). Evaluation of the effect of six sigma management mode in intravenous drug compounding centers. *Guangxi Medicine*.

[20] Ma L., Na M., Pang Y., Zhang L. J. (2020). Evaluation of the application effect of six sigma management model in the management of endoscopic instruments in operating rooms. *China Medical Equipment*.

[21] Chang Y., Jin Y., Guo S. S. (2019). *Integrated Design on Cleaning Instruments of Operating Room and Supply Room and Analysis on Its Application Effect*.

[22] Chand S., Pande P., Prasad A., Anwar M., Dhar Patra D. (2007). Influence of integrated supply of vermicompost and zinc-enriched compost with two graded levels of iron and zinc on the productivity of geranium. *Communications in Soil Science & Plant Analysis*.

[23] Wang Y. J., Hospital Y. C. (2015). The effect of operating room and the disinfection supply center compliance model. *Journal of Taishan Medical College*.

[24] Wang G., Room D. S. (2016). *Discussion on Application of Detail Management in Disinfection and Supply Center*.

[25] Tan Y. L., Si-Tian D. U., Wang X. Y., Cao J. Y. (2018). Value of fine management in the integrated surgical instruments management in operating room and supply room. *China Modern Medicine*.

[26] Gao J., Center D. S. (2018). *Analysis of the Application Value of Evidence-based Nursing Management in the Disinfection Supply Center*.

[27] Cao J. (2017). *Application Value of Detail Nursing in Disinfection Supply Room of Hospital*.

[28] Meng X., Hou X., Cai H., Zhao A. F. (2019). *Clinical Application and Effect Evaluation of Two Kinds Holding Forcep Canister in Different Levels of Clean Operating Room*.

[29] Xiayun L. U., Center D. S. (2017). Application and effect evaluation of hierarchical nursing training in disinfection supply center. *China Health Standard Management*.

[30] Liu Y., Tien Y. H. (2009). Internet research methods: advantages and challenges. *Journal of Nursing*.

[31] Xiulan Y. U., Center D. S., Hospital L. P. (2019). To explore the application of PDCA cycle in nursing management of disinfection supply center. *China Continuing Medical Education*.

[32] Jadhav K. A., Patil A. S., Waghdhare D. S. (2008). Influence of integrated plant nutrient supply on physical and biological properties of soil and yield of okra (*Abelmoschus esculents* L. Monech). *Asian Journal of Soil Science*.

[33] Lin J. (2019). *Application of PDCA Circulation in Nursing Management of Disinfection Supply Center*.

[34] Xiu-Fen H. U., Zhao Y. J. (2017). *Application Value of Detailed Management Model in Nursing Management of Sterile Supply Center*.

[35] Zhao F., Room S. S. (2017). *The Application Value of Detail Nursing in Hospital Sterilization Supply Room*.

